The article "Clustering of Brain Tumor Based on Analysis of MRI Images Using Robust Principal Component Analysis (ROBPCA) Algorithm" was retracted in 2023. Reasons: signs of a paper mill; compromised peer review; unreliable results or conclusions.

# Clustering of Brain Tumor Based on Analysis of MRI Images Using Robust Principal Component Analysis (ROBPCA) Algorithm

**DOI:** 10.1155/2021/5516819

**Published:** 2021-08-31

**Authors:** Ali Hamzenejad, Saeid Jafarzadeh Ghoushchi, Vahid Baradaran

**Affiliations:** ^1^Department of Industrial Engineering, Islamic Azad University, Tehran North Branch, Tehran, Iran; ^2^Faculty of Industrial Engineering, Urmia University of Technology, Urmia, Iran

## Abstract

Automated detection of brain tumor location is essential for both medical and analytical uses. In this paper, we clustered brain MRI images to detect tumor location. To obtain perfect results, we presented an unsupervised robust PCA algorithm to clustered images. The proposed method clusters brain MR image pixels to four leverages. The algorithm is implemented for five brain diseases such as glioma, Huntington, meningioma, Pick, and Alzheimer's. We used ten images of each disease to validate the optimal identification rate. According to the results obtained, 2% of the data in the bad leverage part of the image were determined, which acceptably discerned the tumor. Results show that this method has the potential to detect tumor location for brain disease with high sensitivity. Moreover, results show that the method for the Glioma images has approximately better results than others. However, according to the ROC curve for all selected diseases, the present method can find lesion location.

## 1. Introduction

Imaging techniques used in medicine allow for a relatively accurate diagnosis of diseases without surgery by direct observation of body tissues. Today, many nanotechnology imaging techniques have been improved. Medical imaging is a technique for obtaining images of body components for medical purposes such as diagnosing or studying diseases. The disease can be treated more successfully; that is, the patient's treatment is faster and better with fewer problems and pain and lower costs. Another goal of imaging is to examine the disease's progression and the effectiveness of the treatment [1, 2].

In most literature algorithms for the clustering and classification of MRI, brain MRI is classified by several methods. In [3], the two-dimensional wavelet transforms (DWT) and the Principal Component Analysis (PCA) were employed for feature extraction. The classification they utilized included normal and abnormal brain MR [4]. Chaplot et al. [5] used an approximate two-dimensional subband DWT in MRI images of the brain as new features in the research, in which Daubechies filters were used as a filtering fraction. They considered Alzheimer's disease abnormal. Their studies found that SVM has better results with radial base function and the polynomial core than linear neural networks and SVM [5]. Hackmack et al. [6] (2012) used multidimensional complex wavelet transformations to use MRI images of the brain and then SVM linearly determined whether the brain is multiscale or healthy. The results show that low-frequency scales contain more information than high-frequency values [6]. El-Dahshan et al. [7] used an approximate two-dimensional DWT subband of brain-magnetic MRI in 2015 to compute the feature vector. In their research, Maitra et al. (2008) employed Slantlet deformation, which utilizes its improved DWT variant to obtain the related properties of the MRI of the brain. The fuzzy C-meaning tool was utilized to evaluate brain MRI to determine a natural individual or Alzheimer's disease depending on the features of the image histogram [8]. To distinguish the brain's MRI from a T1-T2 weight, Ramathilagam et al. [9] used a c–means updated algorithm. The authors recommended repeating the dist-max algorithm using the dist-max default algorithm before implementing the algorithm since the c-means standard factor is extremely sensitive to the noise-induced region during extraction [9]. Another study by Lehmann et al., 2017, deals with healthy Alzheimer's patients in the mild and moderate stages of the disease. In this study, 39 different EEG signal features were recorded for individuals with rest and closed eyes. Different classifiers were used to compare differentiating methods of Alzheimer's patients from healthy people [10–12].

In a Kim et al. study, Alzheimer's diagnosis is based on the EEG signal of people employing genetic algorithms and neural networks. The ability to distinguish patients with Alzheimer's from the moderate stage of stable people with a reliable 82 percent of the EEG signal was one of the noteworthy points in this research [13]. An entropy estimate measured the relation of EEG signal disorder to stable individuals with brain tumor patients. In this study, it has been shown that in patients with moderate to severe moderate-to-severe brain tumors, the degree of EEG entropy disorder decreases significantly, most of which are observed in P3 and P4 canals. The findings suggest that low-frequency patients have a more robust power range than normal individuals with low EEG signals, such as the delta and theta bands [14, 15].

Metaheuristic optimization algorithms have become increasingly appealing in recent studies. Metaheuristics are used to identify high-quality solutions to a rising variety of complicated real-world problems, such as combinatorial ones because they can address multiple-objective multiple-solution and nonlinear formulations [16–20]. Optimization methods are at the basis of a variety of vital activities, and they can be applied to a variety of image segmentation problems in medicine [21–25]. There are some optimization methods based on metaheuristic algorithms that can be used for feature extraction in image processing [26–31]. According to methods, Nowinski et al. used the GWR method for the brain's detection. The results show that GWR-based analysis is useful for describing the natural brain, determining areas of interest, and determining healthy age [32]. Haegelen et al. image patterns of T1 weight and T2 were investigated for magnetic resonance imaging with a mean MR image of 57 patients with Parkinson's disease. Animals were better registered than SyN on the left thalamus and better than the right-thalamus patch-based approach [33]. In 2016, Zacharaki et al. studied machine learning algorithms that automatically recognize the related characteristics and are desirable for distinguishing a brain tumor [34]. A research was completed by Fritzsche et al. [35] of 15 brain tumor patients, and of 18 MCI patients, ten were stable for three years, and eight were stable for 15 healthy patients for three years. The diagnosis is also increased with the examination limited to the left brain hemisphere (83.3% accuracy, sensitivity 70%, and 100% attribute). Manual procedures and manual volumes were 66.7% (100.4%) and 72.2% (60.60% 87.5%), respectively [35]. Zarei et al. reviewed the structural tensor scans of MRI scans from 16 patients with AD and 22 healthy volunteers [36]. Using morphometric MRI imaging, Devanand et al. [37] analyzed the local adjustments of the hippocampus, Parahipokamp grains, and entorhinal cortex in determining the conversion from the moderate cognitive disability of MCI to brain tumor of AD [38]. In CT images, such as poor borders, touching organs, and heterogeneity of the liver, Ranjbarzadeh and Saadi proposed a method to resolve liver and tumor segmentation problems. For improved edge extraction, they used the Eight Directional Kirsch filter [39]. In other work, they proposed an algorithm based on the study of the influence of speckle noise on the extended histogram in the speckle noise corrupted image [40]. A new robust algorithm for brain disease classification has been introduced by Hamzenejad et al. The empirical results showed that, while requiring a smaller number of classification attributes, the proposed algorithm obtained a high classification rate and better practices than algorithms recently introduced [41]. Moreover, other research related to brain tumor are RPCA [42] and Optimized Quantum Matched-Filter Technique [43]. Also, biological uses of machine learning are prevalent, for instance, diagnosis of gastric cancer tumor [44], foot fatigue [45], lung tumor [46], tuberculous [47], thyroid nodules [48], Parkinson [49], and paraquat-poisoned patients [50].

In this paper, we used the robust PCA algorithm to cluster MRI images pixel automatically. We used five brain diseases to determine tumor location. The results are compared with fuzzy C-means (FCM) method based on performance analysis criteria.

## 2. Methods and the Material

### 2.1. Robust Principal Component Analysis (Robust PCA or ROBPCA)

One of the essential straight linear algebra results is the analysis of principal components as the nonparametric and straightforward approach is to derive meaningful details from confounding sets. The transformation of the PCA is obtained by decreasing the least-squares error, assuming that the vector of properties is *X* ∈ *R*^*d*^ (*d*-dimensional space), then the space of the reduced features. *Y* ∈ *R*^*h*^. If the vector of properties is *X* ∈ *R*^*d*^, then, the least-squares error can be in the form of

(1) $$\begin{array}{c} \text{MSE}=E\left[{\left\|x-\hat{x\left(r\right)}\right\|}^{2}\right], \end{array}$$

where *x* is the input vector of information, and $\hat{x\left(r\right)}$ is the decoding function for transforming *r* to *x*. In PCA, we are looking for a conversion that obtains the least-squares error, which means the following conversion is desired.

(2) $$\begin{array}{c} T_{D}=\arg\min\left\{MSE\right\}=\arg\underset{\text{r}}{\min}\left\{E\left[{\left\|x-\hat{x\left(r\right)}\right\|}^{2}\right]\right\}. \end{array}$$

It means that we want to find the *r* vector values so that the MSE is as minimal as possible. As mentioned, the PCA is aimed at identifying a linear *T* transformation that generates the least-square error and improves the maximization of this linear $T^{T}\text{ co}{\text{v}}_{x-\hat{x}}T$ transformation in which $\text{co}{\text{v}}_{x-\hat{x}}\;$ is the data covariance matrix with an average of *x*-zero. The PCA then resolves the particular problem, and the *T*-matrix is formed by the vector of unique features of the linear transformation columns. The information is illustrated in the lower dimension $Y=\left(x-\hat{x}\right)$, namely, *Y*. According to the above, MSE has at least *d* − *h* value; that is, a particular large vector corresponding to multiple eigenvalues should be taken to reduce the dimension or the category objective for the minimum MSE. Here, it is necessary to address some of the covariance matrix properties because the main problem is to find the particular values of the covariance matrix. For example, in three dimensions, the covariance matrix is as follows:

(3) $$\begin{array}{c} C=\left(\begin{array}{ccc} \mathrm{cov}\left(x,x\right) & \mathrm{cov}\left(x,y\right) & \mathrm{cov}\left(x,z\right)\\ \mathrm{cov}\left(y,x\right) & \mathrm{cov}\left(y,y\right) & \mathrm{cov}\left(y,z\right)\\ \mathrm{cov}\left(z,x\right) & \mathrm{cov}\left(z,y\right) & \mathrm{cov}\left(z,z\right) \end{array}\right). \end{array}$$

Robust PCA's primary goal is to obtain components that do not affect the outliers, and a powerful covariance estimate matrix has replaced the covariance matrix.

If the primary data of the problem is a matrix *n* × *p* or *X* = *X*_*n*,*p*_, *N* is the number of observations, and *p* specifies the number of variables. The ROBPCA method includes the following three steps:

**Step 1 .**

The data in its preprocessing mode is placed in smaller spaces to a maximum of *n* − 1.

**Step 2 .**

The initial covariance matrix *S*_0_ is created, and the number of components *k* maintained in the sequence is used, which is the product of the *k*-dimensional space in which the data apply. After placing the data in the designated spaces, the dispersion matrix of *k* is the eigenvalue of *l*_1_, ⋯, *l*_*k*_. Eigenvectors are the main component of a powerful problem. The *k*-dimensional component is the *k*-dimensional space decomposition problem that is decomposed from the original *p*-space, which by putting together all the eigenvectors of the matrix *p* × *k* or *P*_*p*,*k*_ . The variable vector *p* determines the estimate. Also, $\hat{\mu }$ is known as a powerful center. Ranks obtained as *n* × *k* matrices from the data or *T*_*n*,*k*_  are specified as follows:

(4) $$\begin{array}{c} T_{n,k}=\left(X_{n,p}-1_{n}{\hat{\mu }}^{T}\right)P_{p,k}, \end{array}$$

where 1_*n*_ is unit diagonal matrix. Also, *k* produces a powerful factor component of the powerful *S* dispersion matrix as much as *p* × *p* with the *k* rank as follows:

(5) $$\begin{array}{c} S=P_{p,k}L_{k,k}P_{p,k}^{T}, \end{array}$$

where *L*_*k*,*k*_ is a diagonal matrix of diameters of eigenvalues *l*_1_, ⋯, *l*_*k*_. The ROBPCA method, like the CPCA, is perpendicular to the spatial and permutable method as if the transformation or rotational transformation (rotation and reverse) is applied to it. Power centers also move or rotate, while ranks remain constant under these transformations. *A*_*p*,*p*_ is a fully ranked orthogonal matrix *A*^*T*^ = A^−1^. Then, *μ*_*x*_ and *P*_*p*,*k*_ are the ROBPCA centers and loading matrix orthogonal data, respectively. Consequently, the converted centers and the scanning matrix are, respectively, equal to *XA*^*T*^ + 1_*n*_ *v*^*T*^ = *Aμ*_*x*_ + *v* and *AP*. Also, ratings after the conversion are fixed as follows:

(6) $$\begin{array}{c} T\left(XA^{T}+1_{n}v^{T}\right)=\left(XA^{T}+1_{n}v^{T}-1_{n}{\left(A{\hat{\mu }}_{x}+v\right)}^{T}AP=\left(X-1_{n}{\hat{\mu }}_{x}^{T}\right)P=T\left(X\right)\right.. \end{array}$$

In all ROBPCA methods, two goals are considered: (a) find a linear combination of variables, even for outlier data; (b) find the type and number of an outlier. The different types of outliers are shown in Figure 1. In this figure, the mapping of data based on robust PCA is depicted. The surface is the 2D PCA space such that data is distributed on it and is fitted by two principal components. Regarding the position of the data, the data points are belonging to such leverages.

The number of levers is defined as follows;

1. *Regular Observation or Regular Leverage*. Refers to data in a homogeneous group in the PCA space
2. *Good Leverage*. Refers to missing or missing data from the original data in the PCA space, such as points 1 and 4
3. *Orthogonal Layer*. Refers to data perpendicular to the PCA space, which is not detectable in the data itself, such as point 5
4. *Bad Leverage*. Data is provided perpendicularly to the PCA space or away from the original or regular data, such as points 2 and 3

A diagram or layer map must be drawn up to detect regular observations with three outliers for high dimension data. The horizontal axis of the diagonal detection layer is the distance between the score distance (SD) and the vertical axis of the orthogonal distance (OD) defined as follows:

(7) $$\begin{array}{c} \text{S}{\text{D}}_{i}=\sqrt{\overset{k}{\underset{j=1}{\sum }}\frac{t_{ij}^{2}}{l_{j}}}. \end{array}$$

The rank *t*_*ij*_ is obtained from the matrix *T*_*n*,*k*_. If *k* = 1, then, SD is equal to the standard score of *t*_*i*_/√*l*_1_. Also, OD is defined as follows:

(8) $$\begin{array}{c} \text{O}{\text{D}}_{i}=\left|\left|x_{i}-\hat{\mu }-P_{p,k}t_{i}^{\prime }\right|\right| \end{array}$$

The *i*-th observation is given as the vector *x*_*i*_ (*p*-variable). Also, *t*_*i*_′ is equal to *i*-th row of the matrix *T*_*n*_. For the separation of an outlier, the horizontal line $\sqrt{\chi_{k,0.75}^{2}}$ for *k* > 1, $\pm \sqrt{\chi_{1,0.975}^{2}}$ for *k* = 1 because the square of the Mahalanobis's decentralization for the data with a normal distribution, it is difficult to determine the vertical cut-off line because there is no information on the distribution of the perpendicular.

## 3. Results and Discussion

### 3.1. Dataset

In this article, we used five brain disorders to apply the proposed approach. The dataset includes Alzheimer's, glioma, Huntington, meningioma, and sarcoma. Such images of diseases include MRI photographs from the repository of Harvard Medical School [51]. All images come from *T*2-weighted MR brain images in the axial plane and have 256 × 256 pixels. Each image is processed separately and analyzed in an unsupervised technique [52].

### 3.2. Results of Proposed Clustering Method

This paper proposes a robust algorithm to determine the tumor location in a magnetic brain image (MRI). MRI image pixels are categorized based on four good, bad, orthogonal, and regular leverages based on the singular value decomposition (SVD) method. The scores obtained from the leverages in the robust PCA algorithm indicate the tumor location. We used five brain diseases, glioma, meningioma, Pick, Huntington, and Alzheimer, to validate this method. Also, ten images such as sensitivity, accuracy, precision, and fallout are recorded. As explained in the method section, the primary purpose of the ROBPCA is to obtain components that do not affect the outlier, and the covariance matrix is replaced by a powerful covariance estimate matrix, which constructs the input image based on four good, bad, orthogonal, and regular. To use ROBPCA, the input parameters of the problem are as follows:

(i) *k*. The number of principal components that will be used in this issue. The number of components is selected using the criteria in Hubert and Engelen [53]
(ii) *Kmax*. Maximum number of principal components to be computed, which is considered a default by 10
(iii) *α*. The robustness parameter is considered to be 0.75 by default
(iv) *h*. The number of anomalies the algorithm has to withstand. Which is obtained from the *n* − *h* equation
  (9) $$\begin{array}{c} h=\left[\alpha *n\right]+1, \end{array}$$
  which *n* represents the sample number. In this case, the value *k* = 0, *k*max = 10, *α* = 0.75, and *h* = 65536. The higher the *α*, the more accurate the calculations for uncontaminated data would be. On the other hand, setting a lower value for *α* would increase the algorithm's robustness in abnormal points. After applying the ROBPCA method, the results are as shown in Figure 2.

Figure 2 shows the graph of pixel clustering results using the ROBPCA method; therefore, each point is the single image's pixels. The results of the ROBPCA analysis include the clustering of pixels into four levers. Two vertical and horizontal cut-off lines separate four leverages. The lower left, lower right, upper left, and upper right levers are regular, good, orthogonal, and bad leverages. The output graph shows the orientation distance (OD) and the distance (SD). The cut-off line for the axis of intermediate distance is 3.338, and the cutting-axis line is 3.0172.

According to the graph of the results of Figure 2, most sample data are located in two orthogonal and regular layers. Regular observations or regular leverage were called data placed in a homogeneous group in the PCA space. The vertical or orthogonal layer was said to be orthogonal to the data that is perpendicular to the PCA space, which is not visible to the data itself.

According to the diagram, 72.7% of data is in the regular lever and 25.3% in the good laver or lexical cluster data that are not directly detected before and 2% in the regular lever. According to the scree plot in Figure 3, four are the best classes using brain images. The scree plot shows the eigenvalue of the covariance matrix of robust PCA. A covariance matrix's eigenvectors and eigenvalues form the “core” of a robust PCA. The new function space directions are determined by the eigenvectors (principal components), and the eigenvalues determine their magnitude. In other words, along the new function axis, the eigenvalues describe the variance of the data. Robust PCA's approach is to perform the covariance matrix's decomposition, a matrix where each element defines the covariance between two characteristics.

The classical PCA method is an approach for reducing the input data's dimension or reducing input variables of features. The robust PCA can reduce the number of features. However, robust PCA is different from PCA. One of the important characteristics of the robust PCA is to separate data into four leverages. This property does not exist in classical PCA. In robust PCA, input data is converted to a single vector then single variables are separated into four leverages. These leverage based on unsupervised clustering property separate data with the same behaviors. Therefore, this method does classical PCA work and applies an unsupervised clustering method to the input data. It can be added that classification and segmentation are machine learning and supervised methods. However, our method is an unsupervised clustering approach. The results of this method can be used in machine learning ground-truth images for the output layer.

After separating the leverage, the image matrix's transformation into the initial image is shown in Figures 4–8. Figures 4–8 show the results of leverage separation for meningioma, glioma, Alzheimer's Huntington, and Pick MRI images. Regarding Figures 4–8, the black parts are in a regular lever and the gray interior parts of the red box representing the vertical lever data. According to the results, tumor location is extracted from bad leverage, and the tiny pixels are removed from the selection. The orthogonal leverage is the complement of regular leverage to construct an original image. In the other use of robust PCA, the bad and good leverages are used as outlier or noise data to clear the input image. However, in this paper, we used outliers to detect tumor location.

### 3.3. Performance Analysis

According to Figure 4, the tumor location of meningioma is approximately well detected. In this case, *α* = 0.7 and colored place from bad leverage have coincided over the original image. In this method, the pixels with the white color using *α* = 0.7 coefficient help to detect optimal location. About glioma and Alzheimer's, this method has the potential for clustering.

To compare with other methods and analyze, we used ground truth images of an automated method of FCM comparison. Therefore, the performance analysis is calculated based on this comparison as follows:

- *True Positive (TP)*. The clustered pixels of the tumor are similar to FCM clustered location
- *False Positive (FP)*. Healthy pixels are detected with discrepancy with FCM
- *True Negative (TN)*. Healthy pixels are detected like FCM
- *False Negative (FN)*. The clustered pixels of the tumor are detected with discrepancy with FCM

The sensitivity of devising the percentages of TP pixels into the sum of TP and FN pixels is defined as follows:

(10) $$\begin{array}{c} \text{Sensitivity}=\frac{\text{TP}}{\text{TP}+\text{FN}}. \end{array}$$

Likewise, the performance analysis's specificity results are the number of false-positive pixels and true negative cases in actual negative cases.

(11) $$\begin{array}{c} \text{Specificity}=\frac{\text{TN}}{\text{TN}+\text{FP}}, \end{array}$$

(12) $$\begin{array}{c} \text{Precision},\text{PPV}=\frac{\text{TP}}{\text{TP}+\text{FP}}, \end{array}$$

(13) $$\begin{array}{c} \text{Accuracy}\left(\text{ACC}\right)=\frac{\text{TP}+\text{TN}}{\text{TP}+\text{TN}+\text{FP}+\text{FN}}, \end{array}$$

(14) $$\begin{array}{c} \text{Fall}-\text{out}\left(\text{FPR}\right)=\frac{\text{FP}}{\text{FP}+\text{FN}}. \end{array}$$

Figure 9 shows the comparison of our presented clustering method with the automated FCM approach. Based on the results of robust PCA, the red pixels show the tumor location. These values are calculated for each disease with ten images. Based on the Pick results, some brain liquid is detected as a tumor that can control with *a* coefficient and Huntington disease because of nonwhite pixels; despite low *α* = 0.6, some worse points are selected. However, with *α* = 0.8, the selection is correct optimally. The sensitivity, fallout, accuracy, precision, and specificity are explained in Table 1. The results illustrated that high sensitivity is demonstrated for glioma brain image; also, this parameter is low for Huntington. It means that this method for Huntington has not high potential to detect tumor location. However, it is perfect for glioma. The specificity and accuracy for all cases are 0.9 and 0.5, respectively. Also, the precision of the approach is nearly is 0.89. The minimum and maximum fallout are shown for Huntington and glioma, respectively. According to the receptive operating characteristic (ROC) curve, we explain that the technique is plausible for all cases. Because all cases have sensitivity greater than fallout, all the cases are above the guess line. Regarding Figure 10, perfect result should have minimum fallout and maximum sensitivity. This method is the potential to detect tumor location for glioma better than others.

## 4. Discussion

Classical PCA is a data-simplification method that uses multivariant databases to lower dimensions for research. It works by calculating the eigenvalues and eigenvalues of a correlation or covariance matrix. In the classical PCA, input data is transformed to a new plane that each coordinates include the greatest variances. Maintaining principal components with the greatest variances and ignoring those with the minor variances contributes to reducing the data dimension while retaining those characteristics of the data set that add the most to its variance.

ROBPCA approach combines projection pursuit with robust scatter matrix estimation and yields more accurate estimates for noncontaminated data and more robust estimates at contaminated data. It is helpful for the analysis of regression data with outliers and multicollinearity. In the case of outliers, the robust PCA produces more concise variants than the nonrobust PCA. Because of the large number of variables in these models, stable PCA solutions to large-scale cointegration models in undersized samples with outliers are of particular interest. In the ROBPCA, the original image is assumed to be contained in an *M* × *N* data matrix *I* = *I*_*M*×*N*_, where *M* denotes the width of the image and *N* is the height. After that, the ROBPCA process is broken down into three main stages. First, the data are preprocessed such that the transformed data are contained inside a subspace of at most *n* dimensions. Following that, a provisional covariance matrix is created and used to choose the number of components *k* that will be preserved in the sequel, resulting in a *k*-dimensional subspace that matches the data well. The data points are then projected onto this subspace, where their position and scatter matrix are robustly determined, and the *k* nonzero eigenvalues are calculated.

The ROBPCA has two aspects: (1) to find certain linear combinations of the original variables that contain the majority of the details, even though there are outliers, and (2) to identify and classify outliers. Therefore, in this paper, we used the second properties of ROBPCA to find tumor location. In the classical PCA, this property does not exist and is used for dimension reduction; however, the ROBPCA clusters data to the leverages. Based on the nature of MRI images, three standard colors are presented, black spots are dominated by empty space, white color illustrates the tumor location, and gray points contain other parts of MRI image such as gray matter (GM), white matter (WM), and cerebrospinal fluid (CSF). Regarding the primary duty of the ROBPCA, the outliers are clustered to three good, bad, and orthogonal leverage, and nonoutlier data is located in regular leverage. This leverage segments the tumor location. The main goal of this paper is to use the clustering properties of ROBPCA to segment MRI images and separate the tumor location as types of outliers. There is no proper performance analysis method for clustering methods because of the unsupervised nature of the method. However, to compare and validate data, we used the results of the FCM method with classification performance analysis. The black points are considered as negative indexes and white pixels (bad leverage) as the positive index. We used 50 images for evaluating the performance of the automated clustering methods. The final performance results illustrate the effectiveness of the presented methods.

## 5. Conclusion

In this paper, a robust algorithm for the determination of tumor location is presented. We use the robust PCA algorithm to cluster image pixels. Robust PCA's results are the clustering of MRI images to four leverages, consisting of regular, orthogonal, good, and bad leverage. In this paper, orthogonal leverage approximately can estimate tumor location. This paper used glioma, meningioma, Pick, Huntington, and Alzheimer's brain diseases to determine the tumor's optimal location. We used ten images of each disease to validate the optimal identification rate. According to the results obtained, 2% of the data in the bad leverage part of the image are determined, which acceptably discerned the tumor. Also, 25.3 percent of the data are located in the orthogonal lever, showing the brain's central and healthy parts. Furthermore, 72.7 percent of the image's data are in the black part that shows other parts of the images. Results show that this method has the potential to detect tumor location for brain disease with high sensitivity. Moreover, results show that the method for the glioma brain images has approximately better results than others. However, according to the ROC curve for all selected diseases, the present method is acceptable.

## Figures and Tables

**Figure 1:** Identify the different types of outliers in ROBPCA.

**Figure 2:** ROBPCA results chart for brain tumor image sample. Upper right side: bad leverage; upper left: orthogonal layer; lower right: good leverage; lower left: regular layer.

**Figure 3:** The scree plot of the robust PCA method.

**Figure 4:** Separation of four levers using the ROBPCA method for meningioma.

**Figure 5:** Separation of four levers using the ROBPCA method for glioma.

**Figure 6:** Separation of four levers using the ROBPCA method for Alzheimer.

**Figure 7:** Separation of four levers using the ROBPCA method for Huntington.

**Figure 8:** Separation of four levers using the ROBPCA method for Pick.

**Figure 9:** The comparison of the presented method with the FCM approach.

**Figure 10:** Receiver operating characteristic (ROC) curve.

**Algorithm 1:** Algorithm robust PCA.

**Table 1:** The results of detection parameters for *α* = 0.8.

	Sensitivity	Specificity	Precision	Accuracy	Fall-out
Meningioma	0.81	0.67	0.89	0.73	0.33
Glioma	0.90	0.5	0.9	0.70	0.5
Alzheimer	0.83	0.67	0.89	0.73	0.33
Huntington	0.42	0.86	0.8	0.63	0.14
Pick	0.50	0.83	0.83	0.66	0.17

## Data Availability

The dataset is available online: http://www.med.harvard.edu/AANLIB/.
